The article "Nursing Teaching Curriculum Setting by Introducing Postcompetency Model under the Vision of Internet Informatization" was retracted in 2023. Reasons: signs of a paper mill; suspected computer-generated content; unreliable results or conclusions; concerns about the data.

# Nursing Teaching Curriculum Setting by Introducing Postcompetency Model under the Vision of Internet Informatization

**DOI:** 10.1155/2022/6164614

**Published:** 2022-09-28

**Authors:** Lan Xiao, Yi Men

**Affiliations:** ^1^Department of Head and Neck Oncology, West China School of Stomatology, Sichuan University, Chengdu, Sichuan, China; ^2^State Key Laboratory of Oral Diseases, West China School of Stomatology, Sichuan University, Chengdu, Sichuan, China; ^3^National Clinical Research Center for Oral Diseases, West China School of Stomatology, Sichuan University, Chengdu, Sichuan, China

## Abstract

The nursing curriculum is to be modernized to improve the student's skills in meeting the recent trends in medical and healthcare fields. The curriculum improvements are based on expert recommendations, authors, and informative data from different web sources. The challenging task is to improve the readability and understandability of the curriculum to real-time standards. Considering the above facts, this article introduces a refined curriculum with Internet information analysis (RC-IIA) method. The proposed method incorporates the distributed Internet, journal, and previous curriculum information within the active nursing syllabus. This prevents repetitions and less-informative content within the active curriculum. Besides, classification learning for knowledge-based representations is used within the curriculum to improve competency. Based on the refined information, a recommendation-based curriculum is preferred for varying information across different standards. The proposed analysis method relies on existing and distributed information across multiple curriculum providers for leveraging the visibility and prolonging the stealth of the nursing curriculum.

## 1. Introduction

A curriculum is a standard-based sequence of experiences containing students' learning skills and practices. The curriculum provides appropriate content and exercise that improves the knowledge of students. The curriculum consists of materials, contents, lessons, and specific learning objectives needed for a teacher to teach a particular course [1]. Nursing courses use various curriculum sets to provide necessary learning opportunities for nurses. The nursing curriculum mostly contains clinical experience, learning activities, and subject-based content that provide a proper plan for faculties [2, 3]. The nursing curriculum is commonly used to train nurses in theoretical and practical ways. Key concepts and important learning skills are included in the nursing curriculum to improve nurses' experience. Teaching nursing curriculum has various types provided to teachers and faculties. Teaching written curriculum contains documented content for teachers and also provides basic topics for the teaching process. The technological curriculum for nursing contains knowledge of equipment and tools that helps to teach the students adequately [4, 5]. The branch of artificial intelligence (AI) known as knowledge representation focuses on representing information about the environment in a form that computers can utilize to accomplish complex tasks like diagnosing a medical problem or having a natural language dialogue. Complex systems can be made easier to design and implement if knowledge representation integrates behavioural findings of how humans solve issues and represent knowledge. Rules and relations between sets and subsets can be automated using logic results in the form of knowledge representation and reasoning. Students that engage in interest-based learning are required to identify personal passions as a means of guiding and leading their educational journeys. The goal of interest-based learning design is to enhance students' innate motivation to learn and to arouse their enthusiasm for education.

The article "Nursing Teaching Curriculum Setting by Introducing Postcompetency Model under the Vision of Internet Informatization" was retracted in 2023. Reasons: signs of a paper mill; suspected computer-generated content; unreliable results or conclusions; concerns about the data.

Informative information is nothing but information that contains helpful and useful details related to particular fields. Informative information improves the performance and knowledge in a particular field [6]. The nursing curriculum contains various information that provides guidelines for nursing students to improve their learning and communicative skills. Informative information is added to the nursing curriculum, providing necessary nursing details to the nursing students [7]. In the nursing curriculum, various subject-related information and practices are included that improve the skills and knowledge of students. Informative information such as professionalism, critical thinking, communication, teamwork, and attitude towards patients is included in the nursing curriculum [8]. Advanced nursing education information and commitment to service-based information are also included in curriculums that enhance the efficiency and effectiveness of nurses. Subject-centred informative information is mostly inserted into a nursing curriculum that provides appropriate details required to improve practical skills. Journals and book details are also included in the nursing curriculum, which contains optimal information about techniques to handle tools and patients [9, 10]. Students' motivation levels and social interaction levels among nursing students are critical to the success of digital tools. As a result, a hybrid learning model that incorporates both on-campus and online learning should be considered, emphasizing the course materials that are most suited to online delivery. These decisions need to be based on the course's specific learning objectives and the subject matter being taught. Distant learning is hampered by the absence of a face-to-face interaction; as a result, educators must devise instructional strategies that promote social connection. Using digital tools for distance learning necessitates a well-structured course to make up for the lack of personal interaction.

The article "Nursing Teaching Curriculum Setting by Introducing Postcompetency Model under the Vision of Internet Informatization" was retracted in 2023. Reasons: signs of a paper mill; suspected computer-generated content; unreliable results or conclusions; concerns about the data.

The correlated curriculum is nothing subject that teaches relationships among each other. A correlated curriculum provides knowledge over co-relation that helps to understand the relationship among each. Internet correlated curriculum plays a vital role in providing knowledge for nursing students [11, 12]. In a curriculum setting, such important and unimportant topics and contents are removed from the nursing curriculum. Internet correlated curriculum setting enhances the performance and reliability of nursing courses that reduce the unwanted stress level of students [13]. Internet correlated curriculum provides various services and functions for nursing students that improve education learning skills and experience. Internet correlated curricula provide certain techniques to learn particular lessons and topics in nursing courses [14, 15]. Internet correlated curriculum improves the quality of education and practical experience of students in nursing fields. Internet correlated curriculum settings provide access control over educational content and information, reducing the time consumption rate in searching journals [16, 17]. The teaching-learning paradigm has recently shifted toward focusing on students. The freedom of choice in education grows stronger. As this ability to choose grows, more time and effort are needed to find the best curriculum for each student's condition and preferences. Individuals' efforts can be minimized, and the proper decisions can be made by providing them with a service that can recommend a preferred curriculum. This work proposes a curriculum recommender system, allowing students to receive guidance before enrolling in classes. This study lays the groundwork for a learner-centred approach to education by offering a customized curriculum right from the start.

## 2. Related Works

Kodera et al. [18] introduced a new behaviour analysing system for nurse trainees. The proposed method is an automatic system that analyses the trainee's behaviour and provides an appropriate set of data for further process. The classification process is used here to find out the exact meaning of the behaviour given by the nurses in healthcare centres. The proposed method increases the accuracy rate in the analysis process, enhancing the system's feasibility and performance.

The article "Nursing Teaching Curriculum Setting by Introducing Postcompetency Model under the Vision of Internet Informatization" was retracted in 2023. Reasons: signs of a paper mill; suspected computer-generated content; unreliable results or conclusions; concerns about the data.

Karimi et al. [19] proposed a machine learning (ML)-based e-school nurse health recognition process. Personalized health-centred e-learning mostly uses ML techniques to identify the health condition of both nurses and students. A deep neural network is used here to understand students' health conditions. Diabetic symptoms are recognized and identified in e-school, which reduces the latency rate in the identification process. The proposed method improves the effectiveness and reliability of the system.

Masuda et al. [20] introduced an informatic nursing curriculum for nursing colleges. An informatics curriculum provides statistical and practical information for nursing students that improves the efficiency level of nurses. Nursing students get health-related data that provide better information for the evaluation process. A separate curriculum is implemented in nursing colleges to provide various details about nursing fields. The proposed informatics curriculum improves the learning skills and awareness of nursing students.

Barrett and Jacob [21] proposed a student success plan (SSP) for nursing colleges that uses a concept-based curriculum. Learning tools are used here to provide access to Internet-based services for the students. A learning navigator (LN) is also used in SSP, which provides appropriate information regarding curriculum and teaching techniques for the faculties. The proposed plan increases the performance rate of faculties in teaching practical sessions for nursing students.

Verkuyl et al. [22] introduced a virtual gaming simulation (VGS) account for nursing education. The proposed method provides an informative curriculum for nursing colleges that improves the performance and feasibility of teaching. The curriculum is implemented based on experiences and practical scenarios that maximize the effectiveness rate in providing services for the students. The proposed method increases the stability of VGS that provide essential teaching skills for nursing faculties.

Tharani et al. [23] proposed a hybrid model for identifying nursing students' mental health competency. Gagne's theoretical framework is used here to determine nursing students' mental health conditions. Features such as communication skills, behaviours, habits, confidence level, and patience rate of nursing students are identified by using a hybrid model. The proposed approach increases the accuracy rate in the identification process, which improves the effectiveness of the system.

Ranse et al. [24] introduced a three-round Delphi design for nursing students. The proposed design is mostly used for understanding the curriculum of nursing courses and provides appropriate meaning for the students. Disaster and accident-related information are added to the nursing curriculum that provides appropriate details for nursing students. The proposed method reduces the stress and pressure rate of nursing students, improving their critical thinking rate.

The article "Nursing Teaching Curriculum Setting by Introducing Postcompetency Model under the Vision of Internet Informatization" was retracted in 2023. Reasons: signs of a paper mill; suspected computer-generated content; unreliable results or conclusions; concerns about the data.

Yang et al. [25] proposed an AHP-Fuzzy comprehensive method for the quality of the simulation evaluation process in the nursing curriculum. A fuzzy comprehensive method is mainly used here to evaluate the teaching techniques of faculties that also increase the quality of the teaching process. The fundamental nursing quality of teachers is evaluated and identified by the AHP-Fuzzy method. The proposed method provides a significant evaluation method for the simulation process that improves the performance rate of the system.

Liaw et al. [26] introduced a scientific approach to translating evidence-based virtual reality into the nursing curriculum. Various strategies are used here to collect information regarding nursing students. Teaching sessions and practices are also included in the nursing curriculum to provide necessary details for nursing students. The science method reduces the analysis process's computation cost and latency rate. The proposed method improves the system's performance, reliability, and effectiveness.

Den Hertog et al. [27] proposed a learning professional knowledge for identifying the experience of Bachelor Nursing (BN) students. The proposed method finds out the quality outcomes of BN students that improve the efficiency and reliability of the system. The proposal also identifies the medium and low-scoring students in BN. The learning approach is used here to provide informative information for a nursing curriculum that enhances the feasibility and quality of nursing students.

Pham et al. [28] introduced a Mental Health First Aid (MHFA) training for nursing students. The proposed MHFA provides necessary skills and techniques in the curriculum for nursing students. MHFA has the appropriate information for nursing students that provide proper first aid skills. MHFA improves the quality of services and feasibility of nursing students. The proposed method improves nursing students' behaviours and mental state and the outcomes of students' stress.

Tseng et al. [29] implemented a clinical simulation scenario in medical-surgical nursing and critical nursing courses. Information technology integrated instruction (ITII) provides various skills and techniques for nursing students. ITII provides an appropriate set of teaching skills and sessions in a nursing curriculum that reduces the critical state of patients in healthcare centres. The proposed method identifies the objective structure of clinical examination (OSCE) scenario in surgical nursing courses.

The article "Nursing Teaching Curriculum Setting by Introducing Postcompetency Model under the Vision of Internet Informatization" was retracted in 2023. Reasons: signs of a paper mill; suspected computer-generated content; unreliable results or conclusions; concerns about the data.

Noh and Kim [30] proposed a self-directed learning program for nursing students using the blended coaching (SDL-BC) technique. The proposed method increases the competency rate of students that provide various clinical practice sessions. Blended coaching is used here for the evaluation process that finds out the effectiveness of self-directed learning of students. Experimental results show that the proposed method improves the implementation of self-directed learning for nursing students. Ngoo et al. [29] proposed NRP benchmark repositories as well as the most recent approaches for solving real-world nurse rostering. This survey is notable for its focus on the rising trends in solution approaches and benchmark datasets. When it comes to dealing with NRPs, meta-heuristics are the most prevalent. In recent years, meta-heuristics has been one of the most common methods for dealing with the NRP. Researchers presently utilize the INRC-I dataset as the most common benchmark to test their methods.

## 3. Proposed Method

The growth of learning resources for education systems fulfils the needs of the current standards and demands in the medical and healthcare fields. The recommendations of the curriculum include service-learning and learning through available resources, that is, online- and offline-based recommendations for their interest in nursing. The service-level learning defines the relationship between the study and service and enables candidates to gain knowledge on practical assistance with courses enhancing the responsibilities of the nursing candidates.  Figure 1 portrays the proposed method.

Classification-based learning is an active learning strategy that makes candidates analyse their responsibilities such as taking care of patients, integrity and dignity of patients, autonomy, and knowledge about handling different types of patients. Curriculum design based on service-learning makes real-time learning taking the candidates closer to meeting the needs of the patients. The recommendation system considers the interest of the learners as well as the domain knowledge of the subjects. It also concerns the changing environment in health care by managing and coordinating the resources to develop specialized nursing candidates to serve patients with utmost care. The recommendation system for nursing candidates enhances the capabilities of the nursing candidate is playing a psychological role in focusing on administrating and maintaining a healthy relationship between patients and healthcare networks. The curriculum of the nursing candidates must be designed comprising the course duration, types of patients and diseases to be addressed, and variations in the treatment according to different stages of the disease with qualitative care ensuring all the needs of the patients. These clinical guidelines should be designed as shown in the following equation:

(1) $$\begin{array}{c} \gamma =C\text{;}\\ \frac{\lambda }{\beta }=\frac{A}{D}\text{.} \end{array}$$

From (1), *γ* is the agreement, where *C* is the percentage of the agreement, *λ* is the evidence level, and *β* represents the grade of recommendation based on which the treatment, diagnosis, and the effects of treatment are monitored. The nursing candidates must be able to handle the psychological behaviour of patients by paying attention to the patients and their families with timely conversations and by providing the appropriate information during the due course of treatment of patients. The anxiety levels of patients are to be monitored; such the abnormalities of the patients can be handled at an earlier stage. The candidates must be trained for active listening and participation in the treatment process by offering a service-based learning curriculum for comprehensive and up-to-date information about the diseases. The curriculum should include effective communication skills so that patients can understand the treatment provided and have a fearless treatment procedure that leads to healthy living. As per the stages of diseases, the candidates must be skilled in handling the symptoms of patients and their anxiety and handling them with the utmost care by organizing workshops and conducting surveys by collecting their feedback from experiences and taking suggestions from patients to establish a healthy relationship between candidates and patients. The curriculum includes training to the candidates from professionals in handling patients at each level regarding the objectives of fulfilling the global vision in the process of identifying the responsibilities in providing care to the patients. Special training must be provided in handling the advanced devices in diagnosing the diseases with the knowledge of their effects on patients and protocols to be followed while undergoing procedures. A curriculum-based framework with a knowledge map is created. It consists of constructing a curriculum for nursing candidates, identifying the relevance between different sources of curriculum, and generating recommendations systems. Initially, a feedback-based set of instructions is collected from nursing candidates and the patients about their experiences. Secondly, a knowledge map is created based on the information from the candidates and patient experiences, on which the degree of relevance is calculated. Finally, the recommendations are made concerning the degree of relevance.

The article "Nursing Teaching Curriculum Setting by Introducing Postcompetency Model under the Vision of Internet Informatization" was retracted in 2023. Reasons: signs of a paper mill; suspected computer-generated content; unreliable results or conclusions; concerns about the data.

Nursing practice in the twenty-first century is challenged by various factors, including an ageing nursing workforce, an increase in the number of elderly and critically ill patients, rising healthcare costs, and a growing shortage of nurses and nurse educators. To keep up with the ever-changing and evolving healthcare environment, nurse educators must constantly evaluate and examine the education curricula, teaching-learning methodologies, and programmes they use to train new professional nurses based on effective nonvisible recommendations.

## 4. Feedback-Based Curriculum

Based on the capability of the candidates, their behaviours towards the interest of the subjects, the overall period of curriculum, and curriculum involving the recent advancements in health care are designed based on the feedback from the candidates and patients with experiences. The ratio of a candidate's capability to the medium of learning is shown in the following equation:

(2) $$\begin{array}{c} \rho_{f}\left(\chi_{i},\alpha_{k}\right)=\frac{\sigma \left(\chi_{i},\alpha_{k}\right)}{\underset{1\leq l\leq N}{O}\sigma \left(\chi_{i},\alpha_{k}\right)}\text{.} \end{array}$$

From (2), *α*_*k*_ represents the medium of learning *k*, *σ*(*χ*_*i*_, *α*_*k*_) is the learning capability of *χ*_*i*_ with a medium of learning *α*_*k*_, and *ρ*_*f*_(*χ*_*i*_, *α*_*k*_)[0,1] is the candidate's preference of interest with a medium of learning. The feedback-based curriculum implication process is represented in Figure 2.

The drafted curriculum is first verified in its visibility, followed by preference and feedback. If all the conditions are positive and linear, then preference is improved. On the contrary, refinement, assimilation, or visibility is verified if any of the conditions fail. These outcomes are analysed such that the feedback maximizes the visibility and recommendation (refer to Figure 2). The time for preference of interest-based learning is calculated as the ratio of the candidate's time taken to learn to the overall time for the medium of learning, as shown in the following equations:

(3) $$\begin{array}{c} \rho_{d}\left(\chi_{i},\alpha_{k}\right)=\frac{\delta \left(\chi_{i},\alpha_{k}\right)}{n*\delta \alpha_{k}}\text{,} \end{array}$$

(4) $$\begin{array}{c} \rho_{d}\left(\chi_{i},\alpha_{k}\right)=\frac{\delta \left(\chi_{i},\alpha_{k}\right)}{\delta \alpha_{k}}\leq n\text{,} \end{array}$$

(5) $$\begin{array}{c} \rho_{d}\left(\chi_{i},\alpha_{k}\right)=1,\frac{\delta \left(\chi_{i},\alpha_{k}\right)}{\delta \alpha_{k}}>n\text{.} \end{array}$$

To meet the demands of today's healthcare industry, education systems are expanding their learning resources based on the curriculum in which students are encouraged to participate in service-learning by using online and offline resources to incorporate the distributed Internet, journal, and previous curriculum. Further, please include the interaction between study and service, defined by service-level learning, which gives students the opportunity to learn about practical through courses that increase the nursing candidates' duties.

The article "Nursing Teaching Curriculum Setting by Introducing Postcompetency Model under the Vision of Internet Informatization" was retracted in 2023. Reasons: signs of a paper mill; suspected computer-generated content; unreliable results or conclusions; concerns about the data.

From the above, Equations (3)–(5) *δ*(*χ*_*i*_, *α*_*k*_) is the time taken to learn for the candidate *χ*_*i*_ with curriculum *α*_*k*_, *δα*_*k*_ is the overall time for medium of learning, and *ρ*_*d*_(*χ*_*i*_, *α*_*k*_) is the preference of interest for the medium of learning, and *n* is the quantity of interest-based on the medium of learning. The ratio of the candidate's capability in different periods' duration to the maximum times of repeated references with the patient's feedback is given by the following equation:

(6) $$\begin{array}{c} \rho_{fdp}\left(\chi_{i},\alpha_{k}\right)=\frac{\delta_{1}\left(\chi_{i},\alpha_{k}\right)+\delta_{2}\left(\chi_{i},\alpha_{k}\right)}{\underset{1\leq l\leq N}{O}\delta_{1}\left(\chi_{i},\alpha_{k}\right)+\delta_{2}\left(\chi_{i},\alpha_{k}\right)+p_{\theta }}\text{.} \end{array}$$

From the above, equation (6) *δ*_1_(*χ*_*i*_, *α*_*k*_) and *δ*_2_(*χ*_*i*_, *α*_*k*_) represent the candidate's learning capability at different periods for the medium of learning. *ρ*_*fdp*_(*χ*_*i*_, *α*_*k*_) is the preference of interest with the medium of learning. The relevance between the medium of learning and the existing curriculum is developed based on relationships between different curricula, that is, the learning medium and the curriculum, within the existing curriculum and the association of curriculum between different courses. The learning medium *α*_*k*_ and the knowledge of the candidate *kχ*_*i*_ are represented as *K∂*. The dependency between the learning medium related to the existing curriculum is represented as *KK,* and the association of curriculum between different courses is defined as*Kς*. A knowledge map is created based on the relevance between the learning medium and the knowledge of the candidate within the curriculum and the association of curriculum that are represented as*K∂*, *KK,* and*Kς*. The learning medium-based knowledge map is defined as shown in the following equation:

(7) $$\begin{array}{c} K_{M}=\left\{u,t\right\}\text{.} \end{array}$$

From Eqn (7), *u* represents node sets in the knowledge map and *t* is the edge between the nodes, where *u*={1,…*ϑ*} and *t*={*t*_*ϑψ*_}. The variable *t*_*ϑψ*_ represents the edge of the nodes *ϑ* and *ψ*. The edge of the sets includes *K∂*, *KK,* and *Kς*. In Figure 3, knowledge map-based classification is illustrated.

The article "Nursing Teaching Curriculum Setting by Introducing Postcompetency Model under the Vision of Internet Informatization" was retracted in 2023. Reasons: signs of a paper mill; suspected computer-generated content; unreliable results or conclusions; concerns about the data.

The preference and feedback are mapped against the classifications (capacity, similarity, interest, and assessment). The KM, as represented in equation (7), relies on a common rate assessment. Depending on the available common feature, the mapping classification is performed. This is required for providing a condition *t*_*vφ*_=1∀ feature >1. The after (unmapped) features are induced for the refined curriculum process; hence, the feedback is augmented (refer to Figure 3). Curriculum creation for nursing programmes necessitates an awareness of the fundamentals of relevant and competency-based curriculum design. In nursing education, curriculum mapping is an evidence-based method of curriculum design that encourages faculty collaboration and quality assurance. Using our large-scale curriculum mapping technique inconsistencies and redundancies in the curricula increase directness.

## 5. Refined Curriculum—Feedback Based

Based on the knowledge map, the recommendation system for the curriculum is designed based on refined factors, namely, feedback, similarity, and refining the candidate are learning capability. The feedback from the learning medium, period for preference of interest-based learning, and the capabilities of the candidate's learning at different periods with the feedback from the experiences of the patients as shown in the following equation:

(8) $$\begin{array}{c} \rho \left(\chi_{i},\alpha_{k}\right)=\omega *\rho_{f}\left(\chi_{i},\alpha_{k}\right)+\mu *\rho_{d}\left(\chi_{i},\alpha_{k}\right)+\eta *\rho_{fdp}\left(\chi_{i},\alpha_{k}\right)\text{.} \end{array}$$

Nursing and medical schools have only partially embraced student involvement, even though it is an established best practice in healthcare services. As a result, some curriculum design has been influenced by students' experiences to better future education. Based on the course and the medium of learning, a score is calculated for the candidates. This scoring matrix is used to identify the similarity between the learning medium and the preference of interest of candidates. The recommendation list based on this scoring matrix is constructed. To improve the accuracy, different combinations of integers were calculated in equation (8) for values of (*ω*, *μ*, *η*) substituted. From these, the highest recommendation accuracy was obtained. The feedback-based classification process for recommendation is presented in Figure 4.

The article "Nursing Teaching Curriculum Setting by Introducing Postcompetency Model under the Vision of Internet Informatization" was retracted in 2023. Reasons: signs of a paper mill; suspected computer-generated content; unreliable results or conclusions; concerns about the data.

The positive and negative feedback inputs are analysed for *φ*_*S*_ and repetition (refer to Figure 4). The correlation between recommendation and accuracy is used for similarity check and relevance-based curriculum output. On the contrary, the repetition for *χ*_*i*_ : to *χ*_*l*_∀ first to last classification is performed. This results in an interest check of the nursing students with an updated curriculum.

## 6. Similarity between Candidates

The similarity between the preference of interest and the course-based learning is identified by calculating the differences in the number of times the candidates learn the courses. The smallest differences in learning the courses and the repetitive number of candidates referring to the same content with the medium of learning are calculated. Professional development practitioners in the field of nursing are urged to incorporate preferred learning methods into their programmes. However, there is enough evidence to draw any firm conclusions regarding the best ways to learn. According to the findings of this study, nursing staff prefer to learn in various ways. According to the findings, learning style preferences were linked to satisfaction, years of experience, and gender. The findings can design and deliver learning experiences that engage participants and help them retain what they have learned.

Based on the behaviour of the candidates, the similarity of the candidate's capabilities is obtained as per following equations:

(9) $$\begin{array}{c} \phi \left(\chi_{i},\chi_{l}\right)=1\text{,} \end{array}$$

(10) $$\begin{array}{c} \phi \left(\chi_{i},\chi_{l}\right)=\frac{1}{\left|\Delta \left(\chi_{i},\chi_{l}\right)\right|},0<\left|\Delta \left(\chi_{i},\chi_{l}\right)\right|<\tau \text{,} \end{array}$$

(11) $$\begin{array}{c} \phi \left(\chi_{i},\chi_{l}\right)=0\text{,}\\ \left|\Delta \left(\chi_{i},\chi_{l}\right)\right|=\tau \text{,} \end{array}$$

(12) $$\begin{array}{c} \phi \left(\chi_{i},\chi_{l}\right)=\frac{1}{\left|\Delta \left(\chi_{i},\chi_{l}\right)\right|-\tau }-1,\left|\Delta \left(\chi_{i},\chi_{l}\right)\right|>\tau \text{.} \end{array}$$

Various tactics are utilized here to acquire information regarding nursing students. Teaching sessions and practices are included in the nursing curriculum to provide vital details for nursing students. The science technique reduces the analysis process's calculation cost and latency rate. The proposed method increases the system's performance, reliability, and effectiveness. From the above equations, Δ represents the difference between the candidate's capabilities for their medium of learning *χ*_*i*_ an d *χ*_*l*_, and *τ* represents the threshold for the difference between the candidate's capabilities. The candidate's similarity is obtained by using the correlation coefficient and the capability of candidates of their preferential medium of learning that is as shown in the following equation:

(13) $$\begin{array}{c} \phi_{S}\left(\chi_{i},\chi_{l}\right)=\varsigma *\phi_{CC}\left(\chi_{i},\chi_{l}\right)+\xi *\phi \left(\chi_{i},\chi_{l}\right)\text{.} \end{array}$$

Equation (13) denotes the combination of the correlation coefficient and the similarity of the candidate's capability. The ratings for the similarity index between the capabilities of the candidates are represented as *ϕ*_*CC*_(*χ*_*i*_, *χ*_*l*_). The refined curriculum from the feedback and the similarity is obtained based on the ratings for a specific medium of learning, which is given by the following equation:

(14) $$\begin{array}{c} \rho_{P}\left(\chi_{i},\alpha_{k}\right)=\underset{\chi_{l}\in neighbor\left(\chi_{i}\right)}{\sum }\phi_{S}\left(\chi_{i},\chi_{l}\right)*\phi \left(\chi_{i},\chi_{l}\right)\text{.} \end{array}$$

The refined curriculum *ρ*_*P*_(*χ*_*i*_, *α*_*k*_) denotes the curriculum according to the medium of learning for a candidate *χ*_*i*_. From the refined curriculum, the recommendation system is designed based on relevance according to the nursing curriculum and the learning medium that is calculated as shown in the following equation:

(15) $$\begin{array}{c} R\left(\alpha_{i},\alpha_{j}\right)=1-\frac{a\Delta \left(i,j\right)}{ο\left(a\right.\left(i,j\right)}\text{.} \end{array}$$

Equation (15) represents the relevance of the candidate's curriculum where *R*(*α*_*i*_, *α*_*j*_) denotes the value for relevance, if the value is greater than it represents that the relevance between the curriculum and medium of learning is greater. It ranges between [0, 1]. A similar relevance-based curriculum drafting process is presented in Figure 5.

The article "Nursing Teaching Curriculum Setting by Introducing Postcompetency Model under the Vision of Internet Informatization" was retracted in 2023. Reasons: signs of a paper mill; suspected computer-generated content; unreliable results or conclusions; concerns about the data.

The candidate capability and similarity measures are used for correlating the relevance and recommendations. These two factors are handled through classification learning due to which preference and information competency are detected. This is required for maximizing the recommendation, and hence, the similarity posts the relevance (Figure 5). Thus, the degree of relevance is obtained on this basis the recommendation to the candidates for a refined curriculum with Internet access information is designed. The performance of the proposed refined curriculum with Internet access information is analysed for its accuracy and recall. The accuracy is given by the following equation:

(16) $$\begin{array}{c} A_{\chi_{i}}=\frac{\left|R_{c}\left(\chi_{i}\right)\cap R_{O}\left(\chi_{i}\right)\right|}{\left|R_{c}\left(\chi_{i}\right)\right|}\text{.} \end{array}$$

Equation (16), *R*_*c*_(*χ*_*i*_) represents the recommendations to the candidate *χ*_*i*_, *R*_*O*_(*χ*_*i*_) represents the preferred medium of learning.

## 7. Discussion

The proposed Rc-IIA is analysed for its performance using the data in [31]. The dataset provides information on student proficiency observed in 2 years for staff appraisals. This information is fetched from 51 district entries of 73,212 students and 6038 staff. For a total of 47 observations, the preference and correlation factors are analysed. When designing classroom and clinical training curriculums for nurses, learning theories serve as the primary guidance. Teachers can apply their understanding of these theories more effectively in various learning circumstances if they are familiar with the general principles. All three dimensions had a common subject of social interaction. Survey data indicated that the majority of students preferred campus-based education and that the pedagogical transition had a negative impact on all aspects of their educational experience. One-third of pupils seemed to favour digital tools for distance learning.

In Table 1, the classifications and other factors (preference, correlation, and visibility) with their changes for 12 observations are tabulated.

The factor changes are based on*χ*_*i*_ to *χ*_*l*_ classifications performed using interest preference. The negative values denote the least feasible input variation, resulting in less significance. As the classification range is high, the feasibility increases; hence, the change of validations is less. For the correlated (similarity) features, the recommendations and preferences are mapped as in Figure 6.

The recommendations and preferences vary with the similarity even in the same observations. Depending on the *φ*_*s*_ and *χ*_*l*_, the variations occur. In Figure 6, the recommendations and preferences for uncommon (left) and common (right) factors are presented. For a common factor [refer to Figure 3], the mapping is provided such that both values are almost the same. The questionnaires for assessing the preference and recommendations are presented in Figure 7.

Based on the questionnaires above, the recommendations and preferences in the curriculum are formulated. This varies from one student to another from which the factors (as in Table 1) are extracted. The extracted factors determine the need for curriculum updates. The classification learning acts as the bridging point in handling preferences, information-centricity, and visibility.

## 8. Comparative Assessment

The comparative assessment for the proposed method is performed alongside the existing AHP-Fuzzy [25], SSP-CC [21], and LKQ-CC [26] methods. The assessment for visibility, recommendation, information refinement, representation ratio, and model latency is provided by varying the *R* and *ρ*.

The article "Nursing Teaching Curriculum Setting by Introducing Postcompetency Model under the Vision of Internet Informatization" was retracted in 2023. Reasons: signs of a paper mill; suspected computer-generated content; unreliable results or conclusions; concerns about the data.

## 9. Visibility Assessment

The comparative assessment for visibility is presented in Figure 8 under different varying factors. The proposed method achieves better visibility by pursuing *γ* the recommendations are improved. The classification relies on content assimilation and repetition check to prevent false feedback. The considerations are based on preference and knowledge map in the successive classification. The common knowledge maps are allocated for preference validation using *ρ*_*d*_(*χ*_*i*_, *α*_*k*_) variants as in equations (2) to (5). This series analyses the variations throughout the time to identify repeated preferences. Therefore, the successive intervals focus on the candidate's interest and *Kς* recommendations for preventing further complexity. In the case of the recommendations, the validations are performed to increase the accuracy in detecting similarity measures. This similarity measure is used for classifying visibility and nonvisibility recommendations. Therefore, the nonvisible recommendations are prevented from providing feedback in successive sessions. In the contrary case, the candidate's interest and recommendation are validated for their accuracy in maximizing this feature.

## 10. Recommendation Assessment

Figure 9 presents the assessment of the recommended ratio for the varying *ρ*. The proposed method achieves better recommendation by identifying *C* across different feedback observed under varying candidate capability and correlation. This proposed method identifies the interest based on the agreement provided at the end of the assessment. In this process, the knowledge map generates multiple features for improving the similarity measure as presented in equations (9) to (12). In the classification process first, the *χ*_*i*_ and *χ*_*l*_ is identified for improving the accuracy. Pursued in the second classification, the *ϕ*_*S*_-based correlation is performed to improve the recommendations. In the least possible case, the decisions on preference and refinement generate a negative recommendation. This is addressed using a repetition check and knowledge map to identify common preferences. Therefore, the recommendation based on preferences is high in the first classification. In the consecutive classification process, the negative feedback is addressed using previous recommendations and content assimilations, preventing misguidances. This process is repeated until the relevance is improved for different candidate capabilities. Therefore, the varying recommendations for the preferences are improved and sustained using the common knowledge maps.

The article "Nursing Teaching Curriculum Setting by Introducing Postcompetency Model under the Vision of Internet Informatization" was retracted in 2023. Reasons: signs of a paper mill; suspected computer-generated content; unreliable results or conclusions; concerns about the data.

## 11. Information Refinement

The required information refinement is performed using varying conditional assessments such as verification of interest and preference. These two features are estimated using Δ computed from equations (9) to (12). In the consecutive process, the visibility is improved to prevent negative feedback such that correlation is the alternating process in validating the instances. The classification learning identifies the negative/adverse estimations of the above features through |Δ(*χ*_*i*_, *χ*_*l*_)| < *τ* verification. Based on the verification, *ρ*(*χ*_*i*_, *α*_*k*_) is analysed such that *t*={*t*_*ϑψ*_} is the common verification point. The interest preference is validated in the consecutive conditional verification to prevent further information refinement. This includes nonaugmenting content, awaiting further recommendations from the candidates. Based on the varying features and decisions across multiple recommendations and relevance factors, the refinement is provided. The proposed method achieves better refinement by augmenting the additional features and maximizing distinct verification sessions. The *K∂* and *Kς* are the refined association for constructing multiple instances for refinement over the varying conditional verifications. Therefore, the proposed method is said to achieve better refinement for the varying recommendation rate and relevance ratios (refer to Figure 10).

## 12. Representation Ratio Assessment

The comparative assessment for the representation ratio is presented in Figure 11 for the varying recommendation rate and relevance ratio. The proposed method is keen on identifying *δ*(*χ*_*i*_, *α*_*k*_)-based extractions on preference and interest. The preference and interest are knowledge mapped for identifying the common feature. If a common feature exists, then the mapping is performed for (*δ*(*χ*_*i*_, *α*_*k*_)/*δα*_*k*_) > *n* condition else, the condition (*δ*(*χ*_*i*_, *α*_*k*_)/*δα*_*k*_) ≤ *n* is satisfied. Based on the varying relevance factors, the *ρ*_*fdp*_(*χ*_*i*_, *α*_*k*_) is estimated; this estimation is required for improving the refinement such that no negative features are observed. The varying inputs are prevented from influencing the representation under varying features. Therefore, the second classification is purely dependent on *ρ*(*χ*_*i*_, *α*_*k*_) such that the *ϕ*(*χ*_*i*_, *χ*_*l*_)=1 is achieved. Based on the observation, the *R*(*α*_*i*_, *α*_*j*_) is modelled. To maximize this feature, the *A*_*χ*_*i*__ is analysed for preventing nonrecommendation classifications. The classification learning discards the noncondition satisfying events to prevent additional overheads. Therefore, the preventive measures in refinement and content augmentation are streamlined to maximize its visibility and representations. To ensure additional overhead and the provision of high-quality nursing events, researchers found that nurses should be educated based on streamlined content augmentation to provide required explanations concerning visibility and representation through the classification learning process. The findings showed that nurses should emphasize the importance of communication when providing refinement and content augmentation to foster the classification learning process.

The article "Nursing Teaching Curriculum Setting by Introducing Postcompetency Model under the Vision of Internet Informatization" was retracted in 2023. Reasons: signs of a paper mill; suspected computer-generated content; unreliable results or conclusions; concerns about the data.

## 13. Model Latency

The comparative assessment for model latency is presented in Figure 12 for the varying *R* factor and *ρ* ratio. The latency is reduced by avoiding multiple conditional verifications using a knowledge map. The common features are analysed for the capability correlation so that the variations are prevented from distinct observations. The first classification estimates *ρ*_*d*_(*χ*_*i*_, *α*_*k*_) for the distinct refinement at the early stages. In the consecutive classification process, the *δ*_1_(*χ*_*i*_, *α*_*k*_) and *δ*_2_(*χ*_*i*_, *α*_*k*_) are classified for any candidate *kχ*_*i*_ verification. From this point, the knowledge mapping is performed to identify similar and uncommon features. The identified feature is verified for satisfying *ϕ*(*χ*_*i*_, *χ*_*l*_) as in equations (9) to (12) such that correlation is high. Nursing's core purpose is to provide high-quality care based on noncondition satisfying events. Classification learning eliminates occurrences that do not meet the predetermined criteria to save time and effort in the long run. To maximize its visibility, the preventative actions in refinement and content enhancement have been streamlined based on the second categorization. As the correlation is high, the repetition is not required, so the computations are halted. The time required in this case is comparatively less, such as moving on to the relevance factor. The proposed method is reliable in identifying the unsatisfied conditions and variations preventing augmented conditions. Besides, the *ρ*_*P*_(*χ*_*i*_, *α*_*k*_) assessment after the classification improves the relevance preventing content augmentation. Therefore, the proposed method requires less latency compared to the other methods. Tables 2 and 3 present the comparative analysis results for the varying recommendation rate and relevance ratios.

## 14. Conclusion

This article introduced and discussed the process and performance of a refined curriculum with the Internet information analysis method. This method is designed with insight for improving the nursing curriculum competency. The proposed method assimilated content from different platforms such as the Internet, journals, and previous standards. The assimilations are refined based on nursing students' interest and relevance for improving the real-time curriculum standardization. In particular, the repetitions and less-informative contents are refined based on classification learning performed at different stages. The classification outputs are provided with a recommendation based on assessment and feedback. The visibility and assimilation are periodically modified based on the classification to reduce the adverse impacts of the curriculum assessment for the nursing students. For the varying recommendation rate, the proposed method achieves 8.43% high visibility, 9.95% high information refinement, 14.85% high representation ratio, and 10.07% less model latency. In order to ensure patient satisfaction and the provision of high-quality nursing care, researchers found that nurses should tell patients about each application and procedure and provide required explanations concerning treatment through an improved recommendation process. The limitation shows that nurses should emphasize the importance of communication to foster recommendations based on assessment and feedback.

The article "Nursing Teaching Curriculum Setting by Introducing Postcompetency Model under the Vision of Internet Informatization" was retracted in 2023. Reasons: signs of a paper mill; suspected computer-generated content; unreliable results or conclusions; concerns about the data.

## Figures and Tables

**Figure 1:** Proposed method.

**Figure 2:** Feedback-based curriculum implication.

**Figure 3:** Knowledge map-based classification.

**Figure 4:** Feedback-based classification.

**Figure 5:** Similarity relevance-based curriculum drafting.

**Figure 6:** Recommendation and preferences.

**Figure 7:** Sample questionnaires for preferences and recommendations.

**Figure 8:** Visibility assessment.

**Figure 9:** Recommendation assessment.

**Figure 10:** Information refinement.

**Figure 11:** Representation ratio assessment.

**Figure 12:** Model latency assessment.

**Table 1:** Classifications and other factors.

Observation	Classifications	Preference	Correlation	Visibility	Preference change	Correlation change	Visibility change
1	29	0.025	0.015	0.016	−0.001	−0.152	0.032
2	32	0.0230	0.008	0.016	−0.008	−0.810	0.042
	48	0.007	0.023	0.019	0.006	0.293	0.025
4	63	0.006	0.025	0.020	0.008	0.916	0.035
5	39	0.012	0.027	0.012	0.005	0.524	0.024
6	58	0.025	0.036	0.017	0.018	1.524	0.033
7	36	0.053	0.001	0.005	−0.004	−0.896	0.008
8	47	0.023	0.012	0.025	−0.002	−0.163	0.014
9	65	−0.027	0.018	0.023	−0.013	−1.091	0.017
10	42	−0.0021	0.029	0.026	0.006	0.703	0.015
11	32	0.003	0.025	0.021	0.003	0.238	0.016
12	86	0.005	0.008	0.019	−0.015	−1.177	0.016

The article "Nursing Teaching Curriculum Setting by Introducing Postcompetency Model under the Vision of Internet Informatization" was retracted in 2023. Reasons: signs of a paper mill; suspected computer-generated content; unreliable results or conclusions; concerns about the data.

**Table 2:** Comparative analysis for varying recommendation rate.

Metrics	AHP-Fuzzy	SSP-CC	LKQ-CC	RC-IIA
Visibility	0.468	0.599	0.786	0.955
Information refinement (/Verification)	0.095	0.155	0.238	0.382
Representation ratio	51.51	65.02	77.95	96.13
Model latency (ms)	519.41	402.86	289.68	182.1

**Table 3:** Comparative analysis for varying relevance ratio.

Metrics	AHP-Fuzzy	SSP-CC	LKQ-CC	RC-IIA
Visibility	0.459	0.623	0.798	0.963
Recommendation (%)	57.75	64.04	71.31	85.967
Information refinement (/Verification)	0.087	0.161	0.256	0.367
Representation ratio	52.07	67.75	79.51	96.146
Model latency (ms)	537.18	428.28	307.07	167.913

## Data Availability

The datasets generated during and/or analysed during the current study are not publicly available due to sensitivity and data use agreement.
